The article "Modulated Electrohyperthermia: A New Hope for Cancer Patients" was published in 2020. Journal: Biomed Res Int.

# Modulated Electrohyperthermia: A New Hope for Cancer Patients

**DOI:** 10.1155/2020/8814878

**Published:** 2020-11-13

**Authors:** Huda F. Alshaibi, Bashayr Al-shehri, Basmah Hassan, Raghad Al-zahrani, Taghreed Assiss

**Affiliations:** ^1^Faculty of Science Biochemistry Department, King Abdulaziz University, Saudi Arabia P.O. Box 52502, Jeddah 21573; ^2^Faculty of Science Biochemistry Department, Undergraduate Students at King Abdulaziz University, Saudi Arabia

## Abstract

According to the World Health Organization, the prevalence of cancer has increased worldwide. Oncological hyperthermia is a group of methods that overheat the malignant tissues locally or systematically. Nevertheless, hyperthermia is not widely accepted, primarily because of the lack of selectivity for cancer cells and because the temperature-triggered higher blood flow increases the nutrient supply to the tumor, raising the risk of metastases. These problems with classical hyperthermia led to the development of modulated electrohyperthermia (mEHT). The biophysical differences of the cancer cells and their healthy hosts allow for selective energy absorption on the membrane rafts of the plasma membrane of the tumor cells, triggering immunogenic cell death. Currently, this method is used in only 34 countries. The effectiveness of conventional oncotherapies increases when it is applied in combination with mEHT. In silico, in vitro, and in vivo preclinical research studies have all shown the extraordinary ability of mEHT to kill malignant cells. Clinical applications have improved the quality of life and the survival of patients. For these reasons, many other research studies are presently in progress worldwide. Thus, the objective of this review is to highlight the capabilities and advantages of mEHT and provide new hopes for cancer patients worldwide.

## 1. Introduction

Cancer is the second leading cause of death worldwide and is considered a universal public health problem with a large impact on healthcare costs. According to the World Health Organization [1], cancer was responsible for around 9.6 million deaths globally in 2018 (WHO 2018).

Ever since cancer was discovered, researchers have struggled to find the best treatment for this lethal disease. As a result, many types of treatments have been developed, including surgery, chemotherapy, radiotherapy, and, more recently, immunotherapy. Among these modalities, the correct choice for patients varies depending on the type and stage of their disease.

One method known to ancient medical practitioners was oncological hyperthermia. This method was described as the overheating of malignant tissues, either locally or systematically. It was the first known oncological therapy used by Hippocrates [2]. In modern times, this technique was used in 1898 by the Swedish gynaecologist Westermark. Westermark treated cervical cancer by running hot water through an intracavitary spiral tube. He noticed an excellent clinical response. Unfortunately, exposing normal healthy tissue to a high temperature for a long time had unfavourable effects [3], in addition to lacking selectivity and thereby damaging the healthy surrounding tissue. Overheating causes increased blood flow, which increases the delivery of nutrients to cancer cells. Moreover, increased blood flow helps disseminate cancer cells and increases the risk of metastasis [4]. The desire to eliminate these side effects of classical hyperthermia led to the discovery of the electromagnetic heating method. This new paradigm is possible due to modulated electrohyperthermia (mEHT), which makes cellular selection possible [5]. The heterogeneous absorption of energy caused by this technique follows the natural biophysical heterogeneity of the tumor and its surrounding tissue [6]. Consequently, the selectively tuned technique changes the isothermal (homogeneous) heating procedures in conventional hyperthermia.

The article "Modulated Electrohyperthermia: A New Hope for Cancer Patients" was published in 2020. Journal: Biomed Res Int.

This technique is used in five continents and 34 countries, with approximately 400,000 treatments performed each year [6]. However, it is not yet known/used in many other countries.

### 1.1. mEHT Mode of Action

The mEHT technique is based on two principles: (1) it replaces the single temperature concept that was used previously in hyperthermia with energy that is measured in (kJ/kg), returning the technique to the gold standard dose concepts known to radiation oncologists [4]; (2) it selectively delivers this energy into the tumor without affecting the healthy neighbouring tissue [7, 8]. To successfully target tumor cells, the modified metabolic and biophysical conditions of cancer cells allow for selective targeting of the energy [9]. In contrast to normal cells, cancer cells rely mainly on anaerobic glycolysis, regardless of oxygen availability. This phenomenon is known as the “Warburg effect” [10]. The fermentation of glucose by cancer cells results in the production of two ATP molecules rather than the 36 ATP molecules that result from the complete oxidation of glucose in the mitochondria of healthy cells [11]. Many applications take advantage of this fundamental difference, such as positron emission tomography (PET) diagnosis. As a result of the increased glucose uptake, the lactic acid production increases, and other metabolites contribute to a higher proliferation rate in the microenvironment of the cancer cells. The subsequently decreased extracellular pH and “reversed” intracellular pH [12–14] also help identify the cancer cells.

The article "Modulated Electrohyperthermia: A New Hope for Cancer Patients" was published in 2020. Journal: Biomed Res Int.

The basic metabolic differences between cancer and noncancer cells make their electrical recognition possible [15] and include the following characteristics:

- The ability of cancer cells to produce sufficient ATP is low. A large amount of ATP is needed for proliferative energy consumption. Cancer has less ATP for active membrane stabilization by K^+^ and Na^+^ transport; thus, the membrane potentiation weakens [16]
- The cellular membrane of cancerous cells is electrochemically different from normal cells, since they are negatively charged on average [17, 18]
- The composition of membrane lipids and sterols differs dramatically between cancer cells and normal healthy cells [19–21]

As a result of these differences, the membrane permeability of cancer cells is altered. Thus, the efflux of K^+^, Mg_2_^+^, and Ca_2_^+^ ions increases, whereas the efflux of Na^+^ and water transport from the cell decreases. Accordingly, the cell swells, which causes an additional reduction in its membrane potential. Furthermore, as the network of cellular connections (cadherins and junctions) [5] are broken, the cancer cells become autonomic, changing the dielectric properties (growing the dielectric permeability) of the microenvironment [15], while the resistance decreases. All of these factors contribute to the negative polarization of the tumor and an increase in its conductivity, which is used in electrochemical cancer therapy [22, 23].

### 1.2. The Working Principle of mEHT

Using mEHT requires a very simple methodological setup [24] that depends on nonequally heating the target area and concentrating the absorbed energy into the extracellular electrolytes [25]. This technique creates nonhomogeneous heating by increasing the temperature gradient between the intracellular and extracellular liquids. The resulting heterogeneity leads to a change in membrane processes and uses the strong synergy between the electrical and temperature effects [26] to initiate the signalling pathway responsible for apoptosis instead of necrosis [9]. This method also uses a modulated radiofrequency current, which flows through the cancerous lesion where it is automatically focused by the higher current density [6] due to its lower resistance [27]. The cancer cell membranes are electrically isolated by more than one million V/m field strength, directing the current flow mainly into the extracellular electrolytes [28–30]. Together, the conductivity and permeability differences can precisely distinguish the cancer cells from healthy cells [26, 31–34]. One of the expected results is membrane disruption of the electrically selected cells. The action of the electric field on cellular division has been extensively studied by various research groups [35–37]. In contrast to what is observed in simple heating processes, the physiological feedback mechanisms of homeostasis do not limit the effects of the electric field, and the adverse effects caused by the increased blood supply can be reduced. The mEHT process primarily delivers energy into the extracellular liquid, which heats up and creates a slight (1/1000°C) temperature difference between the inner and outer temperatures of the cell. Although this difference appears minor, considering how tiny the membrane layer is (5 nm), the difference in standard conditions is so high that it may reach ∼200,000°C/m [38].

The article "Modulated Electrohyperthermia: A New Hope for Cancer Patients" was published in 2020. Journal: Biomed Res Int.

Among the numerous advantages of using mEHT, the main one is the localisation of the high thermal load to only a narrow and precise region of the plasma membrane of the malignant cell [39], where the lipid rafts, which are in the nanoscopic range, can absorb the major energy load [40]. As studies have shown, the size of these rafts depends on the host cells: 10 to –100 nm [41], 25 to –700 nm [42], or 100 to –200 nm [43]. This nanoscopic focus is similar to radiotherapy, where the main target is the breaks of the DNA strand in radiotherapy and the lipid rafts in mEHT [44]. The size and selection similarity is shown in Figure 1 [45].

Due to the proper selection and the individual adaptation of the treatment, mEHT is highly personalised [46]. Consequently, cellular destruction of the malignancy does not require a high-temperature isothermal spot. This fact has physiological advantages and reduces the adverse effects and hot spots. In conventional hyperthermia, the overheating of the healthy tissues causes a massive number of complaints during the treatment process [47]. In mEHT, the local thermal and nonthermal effects [6] are completed with modulation-induced synchrony [48], and the nonsynchronous pathological patterns are recognised [49], opening up the technique to theranostic possibilities [50]. The nonequilibrium heating does not affect the membrane rafts, but the absorbed energy heats the extracellular electrolyte differently than other electrolyte compartments of the selected malignant cells, creating a heat flow through the membrane into the cytosol. Thus, the heat flow will remain active until an equilibrium is reached, as depicted in Figure 2. This process explains the efficacy and reliability of the treatment [4].

In prior studies, phantom measurements of the thermal effects caused by increased temperatures were taken in chopped meat and the liver of a pig [51]. Importantly, an appropriately elevated temperature was measured in the liver of the anesthetised living pig [52]. A thermal effect appropriate for complementary preclinical applications of chemotherapy [53] and radiotherapy [54] was measured. A clinical trial has also shown an appropriate temperature increase for radiochemotherapy without risk of adverse effects in a human uterus cervix [55], which was an important observation of the enhanced pharmacokinetic processes [56].

The article "Modulated Electrohyperthermia: A New Hope for Cancer Patients" was published in 2020. Journal: Biomed Res Int.

### 1.3. In Vitro Studies Using mEHT

Many researchers have investigated the effects of mEHT on various in vitro cell cultures and in vivo allografts and xenografts. Comparisons have shown significant differences between cells treated with the same temperature through mEHT and conventional hyperthermia [9, 57], even in comparison to other capacitive techniques [58]. These studies highlight the differences between cancer cells and normal cells and the advantage of being able to destroy cancer cells selectively. A remarkable number of in vitro and preclinical studies revealed that mEHT induces apoptosis rather than necrosis that characteristically results from traditional hyperthermia after an equivalent dose and cumulative time at 43°C [59]. This apoptotic process was shown using various methods, including morphology, p53 expression, TUNEL assays, and DNA fragmentation [4]. Various in vitro cell culture studies and in vivo allograft and xenograft studies have also observed and documented the synergy of the electric field (nonthermal effect) and the heat (thermal effects) in the mEHT cell destruction mechanism [26, 60]. Another study by Meggyeshazi et al. (2014) treated a HT29 colorectal cancer xenograft with a single shot of mEHT for 30 min at an average power of 4 W and made comparisons with an untreated group. The results showed a vigorous destruction of the invasive colorectal cancer xenograft with a seven-fold peak at 72 h in the group treated with mEHT compared to the untreated control group. The mEHT treatment also caused a significant elevation of DNA fragmentation, nuclear shrinkage, and an increased number of apoptotic bodies. Furthermore, it caused an increase in both the amount of BAX protein and the release of cytochrome c from the mitochondria to the cytoplasm, indicating that mEHT caused the tumor to undergo apoptosis by activating the caspase-independent apoptosis [61] and caspase-dependent [58] pathways.

The mechanism by which mEHT produces apoptosis is important, leading to damage-associated molecular pattern (DAMP) signals that cause immunogenic tumor cell death (ICD). DAMP signals can stimulate the uptake of tumor antigens by antigen-presenting cells [62]. The process of DAMP signals leading to ICD is well known and explained in other cancer treatments, such as chemotherapy [63]. The ICD mechanism involves the translocation of calreticulin to the preapoptotic cell membrane, where heat shock proteins (Hsp70 and Hsp90) and the release of ATP can be observed at the early stages of apoptosis. This process is followed by the passive release of high-mobility group box 1 (HMGB1) at the late stages [64–68], as shown in Figure 3. Thus, the combination of DAMP signals and cancer antigens can facilitate the maturation of antigen-presenting cells and activate antitumor T-cell immunity [68, 69]. Another mEHT study induced the transcription of Hsp70 and Hsp90 together with other members of the heat shock protein family in a xenograft model by subcutaneously injecting colorectal HT29 cancer cells into the femoral region of Balb/c (nu/nu) mice [62]. Furthermore, an early accumulation of calreticulin on the cell membrane was detected after treatment with mEHT [62]. These findings support the rationale of using mEHT as a supplementary therapy with other cancer therapies, such as chemotherapy and radiation. This finding was also supported by another study by Qin et al. (2014) that investigated the benefits of combining mEHT with dendritic cell (DC) immunotherapy on a squamous cell carcinoma (SCCVII) cancer model. This study found that treating the tumors on the legs of mice with mEHT together with injecting DCs resulted in a significant inhibition of the growth of distant tumors on the chest [70]. The same results were obtained in another study [71] when the researchers detected a vaccine-like behaviour in the mEHT process. After the abscopal processes, rechallenging the same tumor in the animal was unsuccessful. This phenomenon is known as the “abscopal effect,” in which irradiating localised tumors cause shrinking in the target tumors and tumors located far from the irradiated area. Although the mechanism underlying the abscopal effect is unclear, the results of the study conducted by Qin et al. in 2014 suggest that it may depend on the activation of the immune system, which is mediated by T cells via the CD3^+^ and CD8^+^ that were activated in the group treated with both mEHT and DC immunotherapy. Moreover, this group showed a high level of expression of a different heat shock protein (GP96), which plays an important role in the uptake of antigens by DCs [70].

The article "Modulated Electrohyperthermia: A New Hope for Cancer Patients" was published in 2020. Journal: Biomed Res Int.

A systemic tumor-specific immunological response could be a key in successfully treating cancer patients. The tumor microenvironment (TME) triggers the immunological response [72]. The penetrating DC could be matured in the TME or in the lymph nodes and form an antigen-presenting cell (APC). The APC creates CD8^+^, killing T cells prepared for the immune responses [73]. This concept of combining DC-based cancer immunotherapy with radiotherapy was used before to treat cancer patients without particular success [74]. The reasons for this failure are not clear, but it is likely that a satisfactory number of DCs were not available; consequently, the maturation of DC did not produce enough APCs for the CD8^+^. Another explanation may be that the available DCs differentiated into immunosuppressive regulatory forms due to the poor TME and inhibited the activation of T cells, missing a characteristic to block the cancer progression [75]. The search for a solution to this challenge led to adding heat shock proteins and electrogene therapy to improve the efficacy of DC immunotherapy [76]. Although it is not yet clear how to manipulate this therapy to achieve an optimal induction of antitumor immunity, ICD appears to be the main factor in a favourable immunogenic TME [74, 77–80].

A study by Qin et al. that used both DC immunotherapy and mEHT interested the researchers in studying mEHT and its abscopal effect in experimental in vivo models. In addition to the help its ICD production provides in forming APC, another advantage of mEHT is its tumor-selective focus, which does not affect the available immune cells. As a result, they remain intact for the expected immune actions. In one study, a CT26 murine colorectal cancer allograft model was used in a combined DC and mEHT therapy [71]. The researchers found that mEHT significantly induced apoptosis and increased the release of Hsp70 into the extracellular matrix, transporting out genetic information. Moreover, a combined treatment of mEHT and DC immunotherapy significantly inhibited the growth of the tumor and increased the number of leukocytes and macrophages, causing more immune effects. This study concluded that mEHT could produce a positive TME for an immunological chain reaction, improving the success rate of intratumoral DC immunotherapy [71]. The findings of this study were similar and confirmed later in a study by Vancsik et al. (2018), which used the same CT26 murine colorectal cancer allograft model and concluded that mEHT induced apoptosis through the stimulation of caspase-dependent programmed cell death and through the release of stress-associated DAMP proteins. Tumor-specific killer T cells subsequently activated, and tumor destruction continued through the immunogenic cell death mechanism, causing the abscopal effect that was suggested in previous studies [81]. Moreover, the in vitro experiments that studied the abscopal effect of mEHT in vivo studies was also conducted such as the study done by Minnaar which involved phase III randomized human trial of cervical cancer the results of this study support the in vitro results earlier and provided evidence of an abscopal effect associated with adding mEHT to the treatment protocol of these patients [82].

The article "Modulated Electrohyperthermia: A New Hope for Cancer Patients" was published in 2020. Journal: Biomed Res Int.

Another study investigated the molecular mechanism underlying the cytotoxic effects of mEHT on different cell types of hepatocellular carcinoma (Huh7 and HepG2) and found that treating hepatocellular carcinoma cells with mEHT increased the inhibitory effect due to a subset of molecular changes. The molecular changes included the upregulation of septin 4 (SEPT4) and inhibition of G-protein-coupled receptor 64 (GPR64), a key regulator of invasiveness, accompanied by the renewal of cyclin-dependent kinase inhibitor p21. These changes enhanced the apoptotic signalling caused by mEHT. In addition, mEHT inhibited the growth of hepatocellular carcinoma xenograft in nude mice [83].

### 1.4. Clinical Trials Using mEHT in Combination with Other Cancer Therapies

Recently, a comprehensive review was published showing the clinical achievements of mEHT that were mirrored in numerous publications [84]. Many preclinical investigations were successfully followed by clinical trials, as summarised in Table 1. The results of a phase III clinical study [85] showed significant increases in the survival and quality of life [86] of patients with advanced, mostly metastatic uterus cervix tumors. The expected abscopal effect, which was shown in the preclinical phase, was also proven clinically [82]. The resulting immunogenic cell death was a great advantage in treating glioblastoma patients [87]. In particular, complicated malignancies with low expected survival rates (like pancreatic or brain gliomas) have been successfully treated with mEHT (see Table 1). A meta-analysis covering various clinical research groups also demonstrated remarkable results in the treatment of advanced brain gliomas [88]. Importantly, lung malignancies (including both small-cell and nonsmall-cell cancers) can be treated successfully when mEHT is used in combination with conventional treatments (see Table 1). The actual status of mEHT therapy for advanced lung malignancies was reviewed in 2014 [89].

The clinical applications of mEHT fit well with various immuno-oncological therapies, like oncolytic viral treatments [90–92] and checkpoint inhibitors [93]. Clinical studies have continued to investigate the effects of mEHT in trials to prove its safety and efficacy in complementary combination with different conventional cancer therapies. These studies have been performed independently in various countries, including Hungary, Germany, S. Korea, China, Italy, Canada, and Austria. The results obtained from these studies are promising. Those patients with advanced disease undergoing mEHT have enjoyed significantly elongated survival times and an improved quality of life is proven. Considering the large number of mEHT treatments worldwide, evidence-based clinical studies, together with overall market surveillance, have registered only rare adverse effects: erythema (8% of patients) or minor adipose burns (3% of patients). In addition, using mEHT like a vaccination could lead to immune modulation and new tumor therapies [92], breaking the therapy resistance to chemotherapy and biological therapy [94]. Presently, more clinical trials are ongoing on other types of cancer, including advanced breast, ovarian, and pancreatic lesions.

The article "Modulated Electrohyperthermia: A New Hope for Cancer Patients" was published in 2020. Journal: Biomed Res Int.

## 2. Conclusion

The effectiveness of modulated electrohyperthermia as a new hyperthermia method has been shown in numerous studies. Its success derives from nanoscopically heating cancer cells with a high degree of cellular selectivity, which changes the heating paradigm from isothermal homogenous heating to selected cellular heating using the natural heterogeneity of the tumor and its host. In addition, this technique enhances the immune-specific response, which promotes the supporting natural, protective, and defending mechanisms of the human body. [95] Thus, mEHT is a promising therapy that may be used during all phases of cancer treatment in combination with other oncology treatments.

This technique has minimal toxicity and side effects. Clinical studies show that mEHT improves the quality of life and survival rate of patients. Despite the present results, more in vitro experiments and clinical pieces of evidence have to be collected for a broader range of applications and better results. This treatment could give new hope to cancer patients.

## Figures and Tables

**Figure 1:** Principle of mEHT therapy. The principles of mEHT and radiotherapy are similar, targeting nano range-sized parts of the cells to induce destruction this figure was adapted from Szasz A [45].

**Figure 2:** Oncothermia targeting the extracellular electrolytes. Oncothermia delivers its energy mainly into extracellular electrolytes, creating a temperature gradient through the cellular membrane [4]. The thermal gradient action due to nonhomogeneous heating is active, until the thermal equilibrium equalises the temperature; this figure was adapted from Gabriella et al. [4].

**Figure 3:** Schematic representation of the stimulation of immunogenic cell death- (ICD-) treating cells with different ICD inducers, such as chemotherapy, radiotherapy, and mEHT, results in the induction of cancer cells, which leads them to undergo apoptosis. Subsequently, apoptotic cells express damage-associated molecular pattern (DAMP) hallmarks, including the translocation of calreticulin from the endoplasmic reticulum to the cell surface, the release of high-mobility group B1 (HMGB1) from the nucleus, the extracellular secretion of ATP, and the expression of various heat shock proteins on the cell surface. This DAMP signal leads to the activation and maturation of dendritic cells, followed by activating several antitumor immune responses. This figure was adapted from Zhou et al. [124].

The article "Modulated Electrohyperthermia: A New Hope for Cancer Patients" was published in 2020. Journal: Biomed Res Int.

**Table 1:** Clinical trials that used mEHT in combination with other treatments.

No.	Tumor site	Number of patients	Treatment used	Results	Reference
1	Relapsed high-grade gliomas	15	mEHT + alkylating chemotherapy	Tolerable and safe for patients with relapses even with a high escalation of the dose.	[96]
2	Advanced gliomas	12	Chemotherapy + radiotherapy + mEHT	CR = 1, PR = 2, RR = 25%. Median duration of response = 10 m. Median survival = 9 m, 25% survival rate at 1 year.	[97]
3	Relapsed malignant gliomas	24	mEHT	Median survival = 19.5 m, 55% survival rate at 1 year, 15% at 2 years.	[98]
4	Advanced glioblastoma	60	mEHT + immunotherapy	No added toxicity by immunotherapy. Median progression-free survival (PFS) = 13 m. Median follow-up 17 m, median OS was not reached. Estimated OS at 30 m was 58%.	[87]
5	Various brain-gliomas	140	Chemotherapy + radiotherapy + mEHT	OS = 20.4 m. mEHT was safe and well tolerated.	[99]
6	High-grade gliomas	179	mEHT + radiotherapy + chemotherapy	Longstanding complete and partial remissions after recurrence in both groups.	[100]
7	Glioblastoma & astrocytoma	149	mEHT + radiotherapy + chemotherapy (BSC, palliative range)	5 y-OS = 83% (AST) in mEHT vs. 5 y-OS = 25% by BSC. 5 y-OS = 3.5% in mEHT vs. 5 y-OS = 1.2% by BSC for GBM. Median OS = 14 m of mEHT for GBM and OS = 16.5 m for AST.	[101]
8	Advanced hepatocell. carcinoma	21	Chemotherapy + mEHT	PR = 1, CR = 0, SD = 11. Combined therapy was effective, and no major complications were observed.	[102]
9	Refractory hepatocell. carcinoma	22	mEHT + thermo-active agents (TAA) or mEHT without TAA	CR = 1, PR = 0. Median OS = 20.5 weeks. 50% showed evidence of increasing QoL and minimal toxicity.	[103]
10	Small-cell lung cancer (SCLC)	22	Chemotherapy + mEHT	mEHT-enhanced destruction of the cancer cells. Improved the OS of patients, too.	[104]
11	Advanced cervical cancer	236	Random. Phase III chemoradiation alone CHR and mEHT group (mEHT + CHR) [preliminary data]	Preliminary data for the first 100 participants. A positive trend in survival and local disease control by mEHT. No significant differences in acute adverse events or QoL between the groups.	[105]
12	Advanced cervical cancer	38	Chemotherapy ± mEHT	The overall response (CR + PR + SD vs. PD) was significantly greater with mEHT. No complications or extra adverse effects by mEHT.	[106]
13	Advanced cervical cancer	72	Radiotherapy + chemotherapy + mEHT	CR + PR = 73.5%, SD = 14.7%. The addition of mEHT increased the QoL and OS.	[107]
14	Advanced cervical carcinoma	20	mEHT + radiotherapy + chemotherapy	mEHT increased the peritumor temperature and blood flow in human cervical tumors, promoting the radiotherapy + chemotherapy.	[55]
15	Advanced cervical carcinoma	108	mEHT + chemoradiotherapy	The complete metabolic response (CMR) of disease outside the radiation field at 6 m posttreatment shows the abscopal effect, significantly associated with the addition of mEHT.	[82]
16	Advanced cervical carcinoma	206	Random. Phase III chemoradiation alone [108] and mEHT group (mEHT + CHR) [preliminary data]	Compliance to mEHT treatment was high (97% completed ≥8 treatments) with no significant differences in CRT-related toxicity between treatment groups or between HIV-positive and HIV-negative participants.	[86]
17	Advanced cervical carcinoma	202	mEHT + chemoradiotherapy	Six-month local disease-free survival (LDFS) = 38.6% for mEHT and LDFS = 19.8% without mEHT (**p** = 0.003). Local disease control (LDC) = 45.5% with mEHT LDC = 24.1% without mEHT; (**p** = 0.003).	[85]
18	Stage III-IV NSCLC	15	Ascorbic acid (AA) infusion + mEHT	AA safely synergises with mEHT and was well tolerated with no major adverse effects.	[109]
19	Advanced NSCLC	97	mEHT + radiotherapy + chemotherapy	Median OS = 9.4 m with mEHT OS = 5.6 m without mEHT; (**p** < 0.0001). Median PFS = 3 m for mEHT and PFS = 1.85 m without mEHT; **p** < 0.0001.	[110]
20	Advanced NSCLC	311 (61 + 197 + 53)	Radiotherapy + chemotherapy + mEHT	Two centres PFY (**n** = 61), HTT (**n** = 197), control (**n** = 53). 80% (PFY), 80% (HTT) had distant metastases, conventional therapies failed. Median OS = 16.4 m (PFY), 15.6 m (HTT), 14 m (control); first-year survival 67.2% (PFY), 64% (HTT), 26.5% (control).	[89, 111]
21	Advanced NSCLC	44	Chemotherapy + ketogenic diet + hyperbaric oxygen + mEHT	Mean OS = 42.9 m, PFS = 41 m. No problems were encountered due to fasting, hypoglycemia, ketogenic diet, mEHT, or hyperbaric oxygen therapy.	[112]
22	Peritoneal carcinomatosis with malignant ascites	260	mEHT + traditional Chinese medicine (TCM) compared to intraperitoneal chemoinfusion [19]	The objective response rate (OPR) = 77.7% in study group (mEHT + TCM) vs. OPR = 63.8% in the ICI group. The QoL = 49.2% vs. 32.3% in the active and control group. Adverse effect rate (AER) = 2.3% vs. 12.3%.	[113]
23	Advanced rectal cancer	76	mEHT + radiotherapy + chemotherapy	Downstaging + tumor regression, ypT0, and ypN0 was better with mEHT than without. No statistical significance.	[114]
24	Liver metastasis from colorectal cancer	80	Chemotherapy + mEHT	Median OS = 24.5 m, and expected (historical) OS = 11 m.	[115]
25	Various types of sarcoma	13	Radiotherapy + chemotherapy + mEHT	Primary, recurrent, and metastatic sarcomas responded to mEHT. The masses regressed.	[116]
26	Soft tissue sarcoma	24	Chemotherapy + mEHT	Pathological response rate (pRR) = 42% in neoadjuvant chemo-hyperthermia treatment median OS = 31 m.	[117]
27	Advanced pancreas carcinoma	25	mEHT + chemotherapy + ketogenic diet + oxygen therapy	Mean follow-up = 25.4 m, median OS = 15.8 m, median PFS = 15.8 m.	[118]
28	Advanced pancreas carcinoma	26	Chemotherapy + mEHT	SD = 9 (48%), PR = 4 (21%) PD = 6 (31%).	[119]
29	Advanced pancreas	106	mEHT + radiotherapy + chemotherapy	After 3 m, PR = 22 (64.7%), SD = 10 (29.4%), PD = 2 (8.3%) with mEHT after 3 m of the therapy. In group without mEHT in the same time: PR = 3 (8.3%), SD = 10 (27.8%), PD = 23 (34.3%). The median OS = 18 m with mEHT and OS = 10.9 m without mEHT.	[101]
30	Advanced pancreas carcinoma	20	Enzyme-therapy + immunolo-modulation + hormone therapy + mEHT	MedianOS > 10m. Most patients experienced partially excellent improvement of QoL.	[55]
31	Advanced pancreas carcinoma	133 (26 + 73 + 34)	Radiotherapy + chemotherapy + mEHT	Two centres PFY (**n** = 26), HTT (**n** = 73), control (**n** = 34). 59% (PFY), 88% (HTT) had distant metastases, conventional therapies failed. Median OS = 12.0 m (PFY), 12.7 m (HTT), 6.5 m (control); first-year survival 46.2% (PFY), 52.1% (HTT), 26.5% (control). QoL was improved.	[120]
32	Ovarian cancer	19	mEHT with dose escalation	The mEHT treatment was feasible in patients with recurrent or progressive ovarian cancer without any complications.	[121]
33	Metastatic cancers (colorectal, ovarian, breast)	23	mEHT + radiotherapy + chemotherapy	OS and time to progression (TTP) were influenced by the number of chemotherapy cycles (**p** < 0.001) and mEHT sessions (**p** < 0.001). Bevacizumab-based chemotherapy with mEHT had a favourable tumor response, was feasible and well-tolerated in metastatic cancer patients.	[122]
34	Different types of metastatic/recurrent cancers	33	mEHT + radiotherapy	CR = 2 (6.1%), very good PR = 5 (15.2%), PR = 13 (39.4%), SD = 9 (27.3%), PD = 4 (12.1%). Three patients (9.1%) developed autoimmune toxicities. All three patients had long-lasting abscopal responses outside the irradiated area.	[93]
35	Advanced gastric cancer	24	mEHT + chemotherapy + ketogenic diet + oxygen therapy	CR = 22 (88%). Mean follow-up = 23.9 m, mean OS = 39.5 m, mean PFS = 36.5 m.	[123]

The article "Modulated Electrohyperthermia: A New Hope for Cancer Patients" was published in 2020. Journal: Biomed Res Int.

## Data Availability

The clinical trial and in vitro study data that were used in this review are cited within the article.

## Abbreviations

AA: Ascorbic acid
AER: Adverse effect rate
AST: Astrocytoma
C26: Murine colorectal cancer cell line
CMR: Complete metabolic response
CR: Complete remission
DAMP: Damage-associated molecular pattern
DC: Dendritic cell
DFS: Disease-free survival
GBM: Glioblastoma multiform
GP96: Heat shock proteins gp96
GPR64: G-protein-coupled receptor 64
HMGB1: High-mobility group box 1
Hsp70 and Hsp90: Heat shock proteins 70 and 90
Huh7 and HepG2: Hepatocellular carcinoma cell lines
ICD: Immunogenic cell death
LDC: Local disease control
LDFS: Local disease-free survival
mEHT: Modulated electrohyperthermia
NED: No evidence of disease
NSCLC: Nonsmall-cell lung cancer
ORR: Objective response rate
OS: Overall survival
PD: Progressive disease
PFS: Progression-free survival
PR: Partial remission
pRR: Pathological response rate
QoL: Quality of life
SCCVII: Squamous cell carcinoma cell line
SCLC: Small-cell lung cancer
SD: Stable disease
SEPT4: Septin 4
TAA: Thermo-active agents
TME: Tumor microenvironment
TTP: Time to progression.
